The article "Effect of Early Radial Shock Wave Treatment on Spasticity in Subacute Stroke Patients: A Pilot Study" was published in 2022. Journal: Biomed Res Int.

# Effect of Early Radial Shock Wave Treatment on Spasticity in Subacute Stroke Patients: A Pilot Study

**DOI:** 10.1155/2022/8064548

**Published:** 2022-07-20

**Authors:** Stefano Brunelli, Noemi Gentileschi, Barbara Spanò, Luca Pratesi, Alessandra Calvani, Roberta Mucci, Calogero Foti

**Affiliations:** ^1^Santa Lucia Foundation IRCCS, Rome, Italy; ^2^Physical and Rehabilitation Medicine, Tor Vergata University, Rome, Italy

## Abstract

**Background:**

Spasticity is a complication that can start immediately after stroke. Radial extracorporeal shock wave therapy (rESWT) is a physical therapy tool used to manage chronic spasticity. However, the effect of rESWT's early use to treat spasticity after stroke is still not clearly investigated. The aim of this study is to evaluate the efficacy of rESWT in improving poststroke spasticity of the upper limb in patients with a recent onset of spasticity compared to conventional physiotherapy alone.

**Methods:**

40 stroke patients were randomly assigned to experimental (EG) or control group (CG). Both groups underwent two daily sessions of conventional rehabilitation therapy (CRT) 5 days per week; the EG underwent one rESWT session a week for 4 weeks. The modified Ashworth scale (MAS) tested at the shoulder, elbow, and wrist was used as outcome measure. MAS was evaluated at baseline, after 2 and 4 rESWT session, and one month after the last session (follow-up).

**Results:**

No significant differences between groups were found at baseline in terms of age, days from onset of spasticity after stroke, and MAS at each body segment. The sample lost eight drop-out patients. Except for the shoulder MAS values, the EG showed statistically significant lower MAS values already after the second rESWT session compared to CG. This significant difference was maintained until the follow-up. The CG showed a significant increase of wrist spasticity after the second evaluation, while the EG maintained constant MAS values throughout the observational period. The elbow spasticity was significantly higher in the CG at the follow-up evaluation.

**Conclusion:**

The rESWT combined with CRT seems to be effective in avoiding the increasing progression of spasticity after stroke.

## 1. Introduction

Spasticity is a common complication after a stroke. Its prevalence has been reported to be 39% in patients with first-ever stroke after 12 months [1]. The time point of onset of spasticity is extremely variable, but according to Wissel et al., it develops during the first 6 weeks after a stroke in 25% of patients, and it affects the elbow in 79% and the wrist in 66% of cases [2]. The constant contraction of spastic muscles can result in pain, reduction of motor function and general mobility, contractures, and skeletal deformities which limit independence in daily living and motor recovery [3]. The mechanism's underlying spasticity may be due to the hyperexcitable stretch reflexes caused by the imbalance between supraspinal inhibitory and excitatory inputs after the upper motor neuron lesion [4]. Along with the neural mechanism, the rheological modifications of the spastic muscles are well known: increase of stiffness, contracture, atrophy, and fibrosis. These structural modifications involve both contractile proteins (reductions in the length of sarcomeres and loss of skeletal muscle fibers) and connective tissue (accumulation of collagenous connective tissue) [5]. Several studies demonstrate that soft tissue changes in paretic limbs begin early after the immobilization resulting from the acute event [6, 7]. The management of spasticity includes a variety of options: antispasticity drugs, intrathecal baclofen, phenol and ethanol injections, administration of botulinum toxin, physical therapy, rehabilitative exercises, and surgery [8].

The article "Effect of Early Radial Shock Wave Treatment on Spasticity in Subacute Stroke Patients: A Pilot Study" was published in 2022. Journal: Biomed Res Int.

The extracorporeal shock wave therapy (ESWT) is a physical modality widely used for the treatment of musculoskeletal diseases [9]. Shock waves are defined as a sequence of single sonic pulses characterized by high peak pressure (100 MPa), fast pressure rise (<10 ns), and short duration (10 *μ*s) and an energy density ranging from 0.003 to 0.890 mJ/mm [10]. Several studies demonstrate efficacy of ESWT in spasticity reduction in the chronic phase after a stroke and in improving functionality of upper [11, 12] and lower limb [13, 14]. To date, there is no consensus on the protocol to be used for the treatment of spasticity in terms of frequency and intensity, but most of the studies use low intensity [15, 16] with values between 0.030 and 0.100 mJ/mm^2^ (corresponding to 1.5-5 bar). Furthermore, there is no evidence of an increase in the therapeutic effect with increasing the amount of the number of pulses used for each single session [16]. Moreover, both focal shock waves and radial shock waves were previously used to treat spasticity, and a recent study has shown that the two types of waves are equally effective [17]. The waves of radial ESWT (rESWT) disperse eccentrically from the applicator tip without concentrating the shock wave field in the targeted tissue, reaching a wider area; they are less invasive and cheaper [18]. Side effects are pain, tingling, redness, and superficial hematoma on the skin, but they are relatively rare and transient [19]. A randomized controlled study carried out in 2016 showed the greater efficacy of 3 ESWT sessions compared to the single session for the spasticity reduction [15]. Furthermore, the study of Wu et al. has shown a noninferiority of ESWT compared to botulinum toxin [20]. The aim of this study was to evaluate the efficacy of rESWT on upper limb spasticity in subacute stroke patients. To the best of our knowledge, no studies investigated rESWT targeted to shoulder, elbow, and wrist performed during the early stages of development of spasticity secondary to stroke. We hypothesized that rESWT, started early after the onset of spasticity and associated with conventional rehabilitation therapy (CRT), may be more effective in reducing the increase of spasticity of the upper limb compared to CRT alone.

The article "Effect of Early Radial Shock Wave Treatment on Spasticity in Subacute Stroke Patients: A Pilot Study" was published in 2022. Journal: Biomed Res Int.

## 2. Materials and Methods

The study took place in an Institute for Neurorehabilitation, Fondazione Santa Lucia. We screened all inpatients with recent stroke that were consecutively admitted to our facilities for a period of 16 months, from May 2020 to August 2021.

### 2.1. Inclusion/Exclusion Criteria

Inclusion criteria were as follows: (1) subacute hemiparesis (within 8 weeks from the ischemic or hemorrhagic stroke onset), (2) first-stroke survivors with confirmed brain lesions by tomography or magnetic resonance imaging, (3) adult age, and (4) presence of spasticity at shoulder or at elbow or at wrist with a modified Ashworth scale >1 or more. Exclusion criteria included the following: (1) previous treatments of the upper limb spasticity with botulinum toxin, phenol, and alcohol; (2) contraindications to shock wave treatment (pregnancy, cancer, coagulopathies, pacemakers, and skin pathologies); (3) presence of an unstable medical condition; (4) persons with cognitive impairment or comprehension aphasia; and (5) presence of disabling comorbidities that compromises upper limb function (such as orthopedic or neurological pathologies).

### 2.2. Recruitment, Randomization, and Ethical Approval

The study was designed as a prospective randomized trial with two parallel groups. After recruitment, all participants were randomly allocated (according to a computer-generated centrally located list) either into the experimental group (EG), treated with rESWT and CRT, or into the control group (CG) treated with CRT alone. Detailed information related to the study aims and procedures was provided to the participants, and written consent was obtained. This study was performed in accordance with the Declaration of Helsinki and was approved by the local independent ethics committee (Approval Number: Prot. CE/PROG.768). The project has been registered as “Current Research (Ricerca Corrente)” with the National Ministry of Health and was registered in ClinicalTrials.gov (ID: NCT04365478).

The article "Effect of Early Radial Shock Wave Treatment on Spasticity in Subacute Stroke Patients: A Pilot Study" was published in 2022. Journal: Biomed Res Int.

### 2.3. Outcome Measures

Primary outcome measure was upper limb spasticity evaluated through the modified Ashworth scale (MAS). We calculated MAS changes in each single district of the paretic upper limb: internal rotators of the shoulder (MAS-s), flexors of the elbow (MAS-e), and flexors of the wrist (MAS-w).

Secondary outcomes were as follows: (1) registration of side effects after rESWT and (2) evaluate if there was a difference in the prescription of oral antispasmodic medication (graded as yes/no) between the 2 groups.

The modified Ashworth scale is a 6-point ordinal scale used to assess muscle spasticity, measuring resistance during muscle passive stretching [21]. As in the previous studies, grade 1+ was matched as 2, so the MAS scores range from 0 (no increase in muscle tone) to 5 (limb rigid in flexion or extension) [20].

Assessments were performed at recruitment (T0), one week after the second session (T1), one week after the fourth session (T2), and one month after the fourth session (follow-up: T3) in both groups. All evaluations were conducted by the same clinician; the clinician was unaware of group allocation of the patient. The evaluations were performed in the morning before any CRT session, while the participants were sitting in his/her wheelchair.

The physicians of the inpatient unit not involved in the study were free to prescribe drugs for spasticity management.

### 2.4. Interventions

The EG underwent one rESWT session a week for consecutive 4 weeks. The treatment was administered during the morning session of CRT. Both groups underwent 2 daily sessions of 40 minutes of conventional rehabilitation therapy for 5 days per week. The CRT consists of facilitation of movements on the paretic side, muscle tone and muscle compensations control, strengthening exercises, stretching exercises, kinesio-taping, trunk stabilization, balance training, standing, sitting and transferring task, conventional assisted overground walking, and occupational therapy aimed at recovering autonomy in the activities of daily life [22].

SHOCK MED device SW1352 (EME, Italy) was used for radial shock wave therapy.

Since targeting the myotendinous junction or muscle belly are both effective for treating spasticity [23], the rESWT was applied with a slow movement “forward and backward” on the anterior area of forearm or arm or shoulder, including the hypertonic muscles and the first third of the proximal and distal tendons (Figure 1).

Two thousand (2000) pulses, 1.5 bar, and frequency of 10 Hz were used to treat each muscular district (shoulder, arm, and forearm). Considering that there is no agreement in the literature on which protocol is the best [24], we have chosen these parameters based on our clinical experience/expertise.

The article "Effect of Early Radial Shock Wave Treatment on Spasticity in Subacute Stroke Patients: A Pilot Study" was published in 2022. Journal: Biomed Res Int.

### 2.5. Statistical Analysis

Continuous variables are reported as mean ± standard deviation. Categorical variables are reported as frequency and percentage. At baseline, between-group differences in age, sex, stroke duration, and MAS were tested using either the Mann-Whitney *U*-test or *χ*^2^ test according to the level of measurement. Change values for the outcome measures were calculated by subtracting the baseline (T0) data from the time points' (T1, T2, and T3) data. To analyze between-group improvement, the Mann-Whitney *U*-test was used.

The within-group effects (i.e., the difference in the outcome measures observed between baseline (T0) and time points (T1, T2, and T3)) were examined by employing the Wilcoxon signed-rank test. We also report the *Z*-score to represent the within-group effect size.

For the outcomes, to avoid the type I error, Bonferroni's correction was applied (*p* value threshold *α* = 0.05/3 = 0.02).

Statistical analyses were carried out using IBM SPSS, version 21.0 (SPSS Inc., Chicago, IL, USA).

## 3. Results

One hundred seventy-five patients with stroke were evaluated in the enrolment period, all of which were admitted into our rehabilitation facility after being transferred from an acute care department. Out of these patients, 40 met the inclusion criteria and were enrolled in the study. There were 8 drop-outs, 3 for CG, and 5 for EG, as shown in Figure 2.

Only the patients (15 EG + 17 CG) that completed the therapy program (CRT or CRT/rESWT) and all clinical evaluations were included in the statistical analysis. Due to COVID-19 problems, two patients in the EG missed the T3 evaluation and were excluded.

Patients' demographic and clinical results at baseline (T0) are shown in Table 1.

EG and CG participants were well matched for age, sex, stroke type, hemispheric stroke side, time from stroke to admission in our inpatients facilities, and time since onset of spasticity. No significant differences between groups were found for any of the outcome measures at baseline (T0).

Table 2 shows the measured outcomes at each time points and change in values, expressed as change between T0 and the respective measurement (T1-T0, T2-T0, and T3-T0) and the between-group statistical results. When comparing EG and CG groups, a significant difference, was observed at T1 in MAS-e and in MAS-w; at T2 in MAS-e and in MAS-w; and at T3 in MAS-s, in MAS-e, and in MAS-w. Conversely, no significant differences between groups were found for MAS-s change values at T1 and T2.

Table 3 shows outcome results at different time points and the within-group differences. With regard to within-group changes, in the EG, no significant changes from baseline (T0) measurements (MAS-s, MAS-e, and MAS-w) were observed at any time point (T1, T2, and T3).

The article "Effect of Early Radial Shock Wave Treatment on Spasticity in Subacute Stroke Patients: A Pilot Study" was published in 2022. Journal: Biomed Res Int.

In the CG, a significant increase was found in MAS-w at T1; in MAS-e and MAS-w at T2; and in MAS-s, MAS-e, and MAS-w at T3.

Then, no significant increase was found in MAS-s and in MAS-e at T1 and/or in MAS-s at T2.

Regarding the secondary aims of the study, during the study, no adverse events were encountered. One patient of EG and 9 patients of CG were treated with oral antispasmodic medication.

## 4. Discussion

This study was aimed at evaluating the effects of 4 monthly sessions of rESWT on the treatment of poststroke spasticity at the early stage of its onset. The target was the spasticity treatment of the main joints of upper limb: shoulder, elbow, and wrist. To the best of our knowledge, this is the first study that investigates the effect of a treatment with rESWT to manage the spasticity of shoulder, elbow, and wrist in stroke in subacute phase.

The results show that the rESWT can yield significant effect on spasticity in subacute stroke patients. We found that the CG showed a constant increase of MAS values, while in the group treated with rESWT, the mean MAS values were similar among all the enrolment period that means stable grade of spasticity without a significant increase.

In literature, most of the studies investigating the use of ESWT for poststroke upper limb spasticity are targeting patients in the chronic phase. In a recent review, Cabanas-Valdés et al. [24] reported that out of the 16 randomized controlled trials, 14 included stroke patients in chronic phase (>6 months) and 2 included patients in the subacute phase. However, these two studies were focused only on the biceps brachii, and time from stroke was greater than in our sample (more than 45 days for both studies) [25, 26]. The authors observed that both at 2 and 4 weeks after ESWT treatment, the elbow MAS score was significantly lower in the experimental group than in patients treated with sham ESWT [25, 26]. In this study, we observed similar results even for the wrist, with a significant between-group difference (EG vs. CG) already from the second rESWT session (Table 2).

The efficacy of rESWT on elbow spasticity in the chronic phase after stroke was reported by several other authors. Yoon et al. reported a reduction of elbow spasticity immediately after the first ESWT session, and this reduction was kept at the evaluation 1 week after the third rESWT session in a sample of chronic stroke patients whose initial MAS was 2.8 ± 0.7 [23]. Bae et al. reported that the elbow spasticity (MAS = 2.9 ± 0.3) improved immediately after ESWT, but no significant effects were reported at 1 week and 4 weeks after ESWT [27]. Conversely, Li et al. reported that after 1-month follow-up, the change in elbow MAS was still evident in chronic stroke patients treated with five consecutive rESWT at 4-day intervals [28]. In this study, we found that, compared to CG, EG had significantly lower scores of elbow MAS starting at the second rESWT treatment, and this difference was maintained until the follow-up. As mentioned above, the EG did not show a decrease of spasticity, but its MAS value was constant for the 2 months of enrolment period, while the CG showed a statistically significant increase at follow-up evaluation. The lack of reduction of the MAS values in the EG could be related to the low initial MAS mean values (1.71 ± 0.59). This could mean that perhaps rESWT is less effective when MAS is low.

The article "Effect of Early Radial Shock Wave Treatment on Spasticity in Subacute Stroke Patients: A Pilot Study" was published in 2022. Journal: Biomed Res Int.

The effects of rESWT on hemiplegic shoulder have been little studied previously. One study reported its efficacy on pain [29]. Only one study investigated the effects of rESWT on spasticity of the paretic shoulder, reporting a significant reduction in spasticity and in shoulder pain treating the subscapularis muscle [30]. Here, we treated the anterior region of the shoulder considering that the pectoralis major plays a pivotal role in the painful, contracted shoulder [31]. We did not find any significant difference between EG and CG when testing the spasticity of the internal rotators of the shoulder. It should be noted that there was a nonstatistically significant trend to increase spasticity over time in the CG (Table 3). We assume that the shoulder spasticity may have a delayed onset after stroke compared to elbow and wrist, but this assumption needs further investigations.

The main positive result of our early rESWT protocol was the effect on spasticity of the wrist. Already after 2 treatments, we found a statistically significant difference between the CG and the EG. This evidence was maintained after 4 treatments and at follow-up evaluation one month after the last treatment. It should be noted that spasticity remains constant in the EG while progressively increasing in the CG. In literature, the efficacy of ESWT on wrist spasticity was previously reported only in a chronic phase. Dymarek et al. found that a single session of rESWT was enough for reduction of spasticity and improving of trophic conditions of the spastic muscles [32]. Manganotti and Amelio reported that a significant reduction of wrist severe spasticity after one ESWT was maintain at 12 weeks after treatment in 50% of enrolled patients [11]. Later, Daliri et al. confirmed that the improvements on wrist flexor spasticity were maintained 5 weeks after ESWT with the evidence of changes in alpha motor neuron excitability [33], but other studies did not report similar neurophysiological evidence after ESWT [11, 13]. Another supposed mechanism is related to the decrease of changes in soft tissues and muscle contractures do to ESWT-related activation of nitric oxide (NO), which has a positive effect on tissue inflammation [34].

The article "Effect of Early Radial Shock Wave Treatment on Spasticity in Subacute Stroke Patients: A Pilot Study" was published in 2022. Journal: Biomed Res Int.

The currently most accepted hypothesis is that ESWT influences the nonneural component of spasticity, improving myofascial viscoelasticity, muscle stiffness, and connective tissue [26]. Our results demonstrate that rESWT is effective even in the early stages of onset of spasticity when muscle stiffness and connective tissue changes are still limited [5]. Further studies are necessary to understand the different mechanisms of ESWT on spasticity when administered in a chronic or in a subacute phase.

Probably, the modest extent of the spasticity reduction reported in our study, unlike what was reported on the stroke patients in chronic phase [24, 35], could be due to a lower fibrotic component of the spastic muscle in the subacute phase. However, since the aim of early treatment is to prevent its formation, studies involving a long-term follow-up period will be necessary.

Our study has several limitations. First, the small number of participants may affect the generalizability of the study findings. Second, the follow-up time should be extended to a longer time to understand if these results are maintained over time. Unfortunately, we could not evaluate it in this study as the postacute in-patient rehabilitation is limited in time and our patients are transferred to another facility within about 3 months. Third, the control group did not perform sham rESWT sessions as in other randomized trials [13, 32]. Finally, we evaluated spasticity only with MAS which is operator-dependent, without associating electrophysiological studies. However, it should be considered that most of the studies that evaluated spasticity use only this clinical scale.

## 5. Conclusions

The early treatment of upper limb muscular spasticity after stroke with rESWT seems to avoid progression to higher degrees of spasticity and reduce the use of oral antispasmodic medication. Further processing of the data of the sample of this study will be carried out to evaluate whether the early rESWT also has an action on the functionality and pain of the upper limb.

## Figures and Tables

**Figure 1:** Methods of treatment with radial extracorporeal shock waves on the forearm flexors.

**Figure 2:** Flow chart.

**Table 1:** Patients' demographic and clinical results at baseline (T0).

	EG (*n* = 15)	CG (*n* = 17)	Between-group differences
Age (years) ^a^	54.80 ± 17.29	62.18 ± 16.17	*U* = 99.50, *Z* = −1.06, *p* = 0.29^#^
Sex (male/female) ^b^	9/6 (60/40)	10/7 (59/41)	*χ* ^2^ = 0.00, df = 1.00, *p* = 0.95^†^
Stroke type (ischemic/hemorrhagic) ^b^	13/2 (87/13)	12/5 (71/29)	*χ* ^2^ = 1.21, df = 1.00, *p* = 0.27^†^
Hemisphere stroke (right/left) ^a^	9/6 (60/40)	7/10 (41/59)	*χ* ^2^ = 1.13, df = 1.00, *p* = 0.29^†^
Time from stroke to admission in our inpatients facilities ^a^	13.53 ± 6.82	15.29 ± 11.10	*U* = 126.50, *Z* = −0.04, *p* = 0.97^#^
Time from stroke and onset of spasticity (days) ^a^	40.80 ± 21.73	39.24 ± 22.08	*U* = 118.50, *Z* = −0.34, *p* = 0.73^#^
MAS-s ^a^	0.33 ± 0.62	0.29 ± 0.69	*U* = 118.50, *Z* = −0.47, *p* = 0.64^#^
MAS-e ^a^	1.60 ± 0.51	1.59 ± 0.80	*U* = 117.00, *Z* = −0.44, *p* = 0.66^#^
MAS-w ^a^	1.33 ± 1.11	1.18 ± 1.07	*U* = 117.50, *Z* = −0.39, *p* = 0.70^#^

EG: experimental group; CG: control group; MAS: modified Ashworth scale; MAS-s: MAS of the shoulder; MAS-e: MAS of the elbow; MAS-w: MAS of the wrist. ^a^Values are expressed as mean ± SD. ^b^Values are counts (%). ^#^Mann-Whitney *U*-test. ^†^Pearson's *χ*^2^. See text for more details.

The article "Effect of Early Radial Shock Wave Treatment on Spasticity in Subacute Stroke Patients: A Pilot Study" was published in 2022. Journal: Biomed Res Int.

**Table 2:** Value changes of the outcome measures at the different time points and between-group statistical results.

	EG (*n* = 15)				CG (*n* = 17)				Between-group differences
	T0	T1	T2	T3	T0	T1	T2	T3	
MAS-s	0.33 ± 0.62	0.33 ± 0.62	0.40 ± 0.63	0.27 ± 0.46	0.29 ± 0.69	0.71 ± 0.92	0.94 ± 0.97	1.29 ± 1.05	
T1-T0 change values	0.00 ± 0.65				0.41 ± 0.80				*U* = 105.00, *Z* = −1.18, *p* = 0.24
T2-T0 change values	0.07 ± 0.80				0.65 ± 0.86				*U* = 91.00, *Z* = −1.56, *p* = 0.12
T3-T0 change values	−0.07 ± 0.70				1.00 ± 1.17				*U* = 62.50, *Z* = −2.68, *p* = 0.01^∗^
MAS-e	1.60 ± 0.51	1.13 ± 0.74	1.13 ± 0.83	1.07 ± 1.10	1.59 ± 0.80	2.12 ± 0.70	2.35 ± 0.86	2.71 ± 1.16	
T1-T0 change values	−0.47 ± 0.64				0.53 ± 0.80				*U* = 46.50, *Z* = −3.23, *p* < 0.001^∗^
T2-T0 change values	−0.47 ± 0.64				0.76 ± 0.97				*U* = 38.50, *Z* = −3.52, *p* < 0.001^∗^
T3-T0 change values	−0.53 ± 1.06				1.12 ± 1.41				*U* = 47.00, *Z* = −3.09, *p* < 0.001^∗^
MAS-w	1.33 ± 1.11	1.00 ± 0.93	1.00 ± 1.07	1.13 ± 1.19	1.18 ± 1.07	1.94 ± 1.03	2.35 ± 0.93	2.82 ± 1.24	
T1-T0 change values	−0.33 ± 0.82				0.76 ± 0.83				*U* = 40.00, *Z* = −3.50, *p* < 0.001^∗^
T2-T0 change values	−0.33 ± 0.82				1.18 ± 0.95				*U* = 27.50, *Z* = −3.91, *p* < 0.001^∗^
T3-T0 change values	−0.20 ± 1.08				1.65 ± 1.32				*U* = 32.00, *Z* = −3.70, *p* < 0.001^∗^

EG: experimental group; CG: control group; *p* value: between-group difference, Mann-Whitney *U*-test; ∗: significant between-group difference at *p* < 0.02; MAS: modified Ashworth scale; MAS-s: MAS of the shoulder; MAS-e: MAS of the elbow; MAS-w: MAS of the wrist. Change values were calculated by subtracting the baseline (T0) data from the time points' (T1, T2, and T3) data. Change values are expressed as mean ± SD. See text for more details.

The article "Effect of Early Radial Shock Wave Treatment on Spasticity in Subacute Stroke Patients: A Pilot Study" was published in 2022. Journal: Biomed Res Int.

**Table 3:** Outcome results at different time points and within-group statistical results.

		MAS-s				MAS-e				MAS-w			
		T0	T1	T2	T3	T0	T1	T2	T3	T0	T1	T2	T3
EG (*n* = 15)		0.33 ± 0.62	0.33 ± 0.62	0.40 ± 0.63	0.27 ± 0.46	1.60 ± 0.51	1.13 ± 0.74	1.13 ± 0.83	1.07 ± 1.10	1.33 ± 1.11	1.00 ± 0.93	1.00 ± 1.07	1.13 ± 1.19
	Within-group differences^#^	*Z* = 0.00, *p* = 1.00				*Z* = −2.33, *p* = 0.02				*Z* = −1.51, *p* = 0.13			
		*Z* = −0.33, *p* = 0.74				*Z* = −2.33, *p* = 0.02				*Z* = −1.51, *p* = 0.13			
		*Z* = −0.38, *p* = 0.71				*Z* = −1.81, *p* = 0.07				*Z* = −1.15, *p* = 0.25			
CG (*n* = 17)		0.29 ± 0.69	0.71 ± 0.92	0.94 ± 0.97	1.29 ± 1.05	1.59 ± 0.80	2.12 ± 0.70	2.35 ± 0.86	2.71 ± 1.16	1.18 ± 1.07	1.94 ± 1.03	2.35 ± 0.93	2.82 ± 1.24
	Within-group differences^#^	*Z* = −1.89, *p* = 0.06				*Z* = −2.32, *p* = 0.02				*Z* = −2.97, *p* < 0.001^∗^			
		*Z* = −2.43, *p* = 0.02				*Z* = −2.62, *p* = 0.01^∗^				*Z* = −3.27, *p* < 0.001∗			
		*Z* = −2.71, *p* = 0.01^∗^				*Z* = −2.63, *p* = 0.01^∗^				*Z* = −3.21, *p* < 0.001^∗^			

EG: experimental group; CG: control group; ^#^Mann-Whitney *U*-test; ∗: significant difference at *p* < 0.02; MAS: modified Ashworth scale; MAS-s: MAS of the shoulder; MAS-e: MAS of the elbow; MAS-w: MAS of the wrist. Outcome values are expressed as mean ± SD. See text for more details.

## Data Availability

The data used to support the findings of this study are available from the corresponding author upon request.

## Acronyms

rESWT: Radial extracorporeal shock wave therapy
CRT: Conventional rehabilitation therapy
MAS: Modified Ashworth scale
MAS-s: Modified Ashworth scale of the shoulder
MAS-e: Modified Ashworth scale of the elbow
MAS-w: Modified Ashworth scale of the wrist
EG: Experimental group
CG: Control group
T0: Baseline evaluation
T1: MAS evaluation one week after the second rESWT
T2: MAS evaluation one week after the fourth rESWT
T3: MAS evaluation one month after the fourth rESWT.
